The article "A Toxin-Antitoxin Module of Salmonella Promotes Virulence in Mice" was retracted in 2020. Reasons: manipulated images; duplicated images; concerns about the images.

# A Toxin-Antitoxin Module of *Salmonella* Promotes Virulence in Mice

**DOI:** 10.1371/journal.ppat.1003827

**Published:** 2013-12-19

**Authors:** Miguel A. De la Cruz, Weidong Zhao, Carine Farenc, Grégory Gimenez, Didier Raoult, Christian Cambillau, Jean-Pierre Gorvel, Stéphane Méresse

**Affiliations:** 1 Aix-Marseille University, CIML, Marseille, France; 2 CNRS, UMR 7280, Marseille, France; 3 INSERM, U631, Marseille, France; 4 Aix-Marseille University, AFMB, Marseille, France; 5 CNRS, UMR 7257, Marseille, France; 6 URMITE, CNRS-IRD UMR 6236, Marseille, France; University of Utah, United States of America

## Abstract

Toxin-antitoxin (TA) modules are widely prevalent in both bacteria and archaea. Originally described as stabilizing elements of plasmids, TA modules are also widespread on bacterial chromosomes. These modules promote bacterial persistence in response to specific environmental stresses. So far, the possibility that TA modules could be involved in bacterial virulence has been largely neglected, but recent comparative genomic studies have shown that the presence of TA modules is significantly associated with the pathogenicity of bacteria. Using *Salmonella* as a model, we investigated whether TA modules help bacteria to overcome the stress conditions encountered during colonization, thereby supporting virulence in the host. By bioinformatics analyses, we found that the genome of the pathogenic bacterium *Salmonella* Typhimurium encodes at least 11 type II TA modules. Several of these are conserved in other pathogenic strains but absent from non-pathogenic species indicating that certain TA modules might play a role in *Salmonella* pathogenicity. We show that one TA module, hereafter referred to as *sehAB*, plays a transient role in virulence in perorally inoculated mice. The use of a transcriptional reporter demonstrated that bacteria in which *sehAB* is strongly activated are predominantly localized in the mesenteric lymph nodes. In addition, *sehAB* was shown to be important for the survival of *Salmonella* in these peripheral lymphoid organs. These data indicate that the transient activation of a type II TA module can bring a selective advantage favouring virulence and demonstrate that TA modules are engaged in *Salmonella* pathogenesis.

**Authors Summary**

Bacteria have the capacity to rapidly adapt to and survive ever-changing environments. This aptitude is essential for a foodborne pathogen that upon ingestion by a host, and in a short period of time, will switch from a free-living state in the contaminated food to a parasitic existence in a host. During this process, the pathogen has to face various destructive surroundings such as the gastric acid of the stomach, the antimicrobiotic activities of the intestinal milieu, or the host immune defences. This raises the question of how a pathogen achieves this rapid adaptation. Bacteria are capable of regulating their biochemical activity with the help of self-toxins. These toxins are normally associated with an antitoxin that limits their toxic activity. In response to unfavourable environmental conditions, the toxin is rapidly freed from the antitoxin and slows down the biological activity of the bacterium. This makes the bacterium less sensitive to harmful environments. In the present study, we investigated whether the bacterial pathogen *Salmonella* possesses similar self-protecting systems and if they are necessary for virulence. We found that these systems are present in pathogenic species of *Salmonella* and help the bacterium establish an infection.

The article "A Toxin-Antitoxin Module of Salmonella Promotes Virulence in Mice" was retracted in 2020. Reasons: manipulated images; duplicated images; concerns about the images.

## Introduction

Prokaryotic genomes contain toxin–antitoxin (TA) loci that induce cell dormancy in response to various stresses [1], [2]. This is mediated by the toxin components that target essential cellular processes, such as DNA replication, mRNA stability or protein synthesis (for review see [2]). Five types of TA systems have been described. In type I and III, the antitoxin is a RNA molecule that either regulates toxin gene expression (type I) or forms a complex with the toxin protein and inhibits its activity (type III) [3]. The recently described type IV and V systems refer to protein-protein modules in which the antitoxin masks the toxin activity either by interfering with binding of the toxin to its target (type IV) [4] or by cleaving specifically the toxin mRNA (type V) [5]. In type II modules, toxin and antitoxin are proteins that are co-transcribed from an operon. By binding its cognate toxin, the antitoxin blocks the toxin activity. Very often, the antitoxin binds to a palindromic stretch within the promoter region and represses the transcription of the operon. Environmental conditions that favour the degradation of the labile antitoxin raise the level of free toxin and also relieve the expression inhibition of the TA locus. This regulation loop maintains a high level of free toxin as long as the conditions supporting the antitoxin degradation are sustained.

Type II TA modules are widely prevalent in prokaryotes. In 2009, a genomic analysis in 750 complete genomes of archaea and bacteria discovered previously unnoticed protein families that are homologous to toxins and antitoxins of known type II TA and highlighted their exceptional mobility [6]. A comprehensive search on 2181 prokaryotic genomes detected more than 10000 sequences that were grouped within toxin (12) and antitoxin (20) super-families [7]. These systems have been proposed to be beneficial in hostile conditions by favouring persistence [8]. However, the circumstances under which TA modules are activated and support bacterial persistence remain poorly understood.

The article "A Toxin-Antitoxin Module of Salmonella Promotes Virulence in Mice" was retracted in 2020. Reasons: manipulated images; duplicated images; concerns about the images.

A study published in 2005 established that TA modules are abundant in free-living prokaryotes but rare in obligate host-associated organisms [9]. It led to the conclusion that TA modules are stress-response elements that increase the fitness of free-living prokaryotes. However, more recent data reported the presence of TA modules in pathogenic intracellular bacteria [7] and a significant association with the pathogenicity of epidemic bacteria [10]. *Mycobacterium tuberculosis* contains more than 60 TA systems, while the saprophytic *Mycobacterium smegmatis* has only two [9]. *Ricketsia* spp., which are obligate intracellular pathogens, possesses up to 32 TA modules [7] and are capable of inducing host cell death in a TA-dependent manner [11]. Elsewhere it has been established that TA modules can promote the colonization of the mouse bladder or kidneys by an uropathogenic strain of *Escherichia coli* [12]. Hence, there is increasing evidence that TA modules are related to bacterial pathogenicity and involved in host-pathogen interactions.

Salmonellae are Gram-negative bacteria responsible for severe gastroenteritis and systemic infections in humans. These bacteria are widespread and commonly found in the intestinal tract of cold- and warm-blooded animals and in the environment where their association with protozoa such as amoebae is thought to favour persistence and transmission [13], [14]. Salmonellae must therefore have evolved mechanisms to rapidly adapt to the multitude of environmental conditions encountered either as free-living organism or as a pathogen in association with a host. The present study investigated the presence of type II TA loci in strains of *Salmonella* and their possible role in virulence.

## Results

### Identification of type II TA modules in *Salmonella* Typhimurium

Bioinformatics analysis using the RASTA-Bacteria webtool [15] and BLASTP of already identified toxins and antitoxins confirmed the presence of eleven type II TA modules in the *Salmonella enterica* subsp. *enterica* serovar Typhimurium (*S*. Typhimurium) genome, nine located on the chromosome and two in the virulence plasmid (pSLT) (Table 1). They belong to five distinct super-families of toxins (see Table 1) [16]. Two of these modules (STM2954.1N-STM2955.S, STM4032.2N-STM4033) have been previously identified in *S.* Typhimurium LT2 [9], while the *vapBC* locus (STM 3033-STM3034) has been shown to be a bona fide type II TA loci [17]. Of note, we could not establish any correspondence between six other TA modules described in the afore-mentioned study [9] and the other TA modules described herein.

The article "A Toxin-Antitoxin Module of Salmonella Promotes Virulence in Mice" was retracted in 2020. Reasons: manipulated images; duplicated images; concerns about the images.

**Table 1:** Identification and family distribution of *S.* Typhimurium TA loci.

Module (The gene of the operon coding for the toxin is underlined)	Homologue (based on the toxin)	Superfamily	Reference
STM1550-STM1551	*relEB* (*E. coli*)	RelE	[51]
STM2954.1N-STM2955.S	*mazEF* (*E. coli*)	MazF	[52], [9]
STM3033-STM3034	*vapBC* (*E. coli* and *S. flexneri*)	VapC	[17]
STM3516-STM3517	*dinJ*-*yafQ* (*E. coli*)	RelE	[53]
STM3558-STM3559	*phd*-*doc* (*E. coli*)	Doc	[54]
STM3777-STM3778	*relEB* (*E. coli*)	RelE	[51]
STM4030.S-STM4031	*higBA* (*E. coli* and *V. cholerae*)	RelE	[40], [55]
STM4032.2N-STM4033	*higBA* (*E. coli*)	RelE	[9], [40]
STM4449-STM4450	*relEB* (*E. coli*)	RelE	[51]
PSLT027-PSLT028	*ccdAB* (*E. coli*)	CcdB	[56]
PSLT106-PSLT107	*vapBC* (*E. coli* and *S. flexneri*)	VapC	[17]

The genus *Salmonella* comprises two species, *S. bongori* and *S. enterica*. The majority of human infections are caused by various serovars of *S. enterica* while *S. bongori* does not cause disease in mammals [18]. We used BLASTP of *S*. Typhimurium chromosomal toxins and genomic context analyses to examine sequenced genomes of Salmonellae for homologs of these TA systems. Using an in-house R script [19], we performed a hierarchical clustering based on the Euclidean distance for the presence or absence of TA modules in the studied genomes as illustrated in the heatmap in Figure 1A. The clustering of bacteria in the horizontal dendrogram indicates the presence of two main clusters. The first cluster consists of serovars of *S. enterica* subspecies *enterica*, which are associated with warm-blooded host, that have between five and eight of the nine chromosomal TA modules found in *S* Typhimurium (Figure 1A). Interestingly, four of these TA modules are present in all serovars of *S. enterica* subspecies *enterica*. The second cluster comprises subspecies *houtenae* and *arizonae* of *S. enterica*, which infect cold-blooded animals and the non-pathogenic species *S. bongori*. The subspecies *houtenae* and *arizonae* present a low number of modules (two and four, respectively), while none are present in *S. bongori*. These analyses indicate that TA modules detected in *S*. Typhimurium are more prevalent in strains associated with warm-blooded hosts as compared to strains that infect cold-blooded animals. They also suggest a role in pathogenesis since these TA modules are absent from the non-pathogenic species *S. bongori*.

**Figure 1:** Conservation of TA modules across the genus *Salmonella*. (**A**) The toxins of *S*. Typhimurium TA modules were subjected to BLASTP against various *Salmonella* strains. Serovars of *S. enterica* subsp. *enterica* are coloured in red. *Arizonae* and *houtenae* subspecies of *S. enterica* are coloured in blue. The non-pathogenic species *bongori* is coloured in green. All sequences were taken of NCBI and ColiBASE databases. Gene products were clustered according to their presence (black) or absence (light grey). Incomplete modules are indicated in dark grey. (**B**) Genetic organization of the STM4031-STM4030.S and STM4032.2N-STM4033 modules in *S*. Typhimurium chromosome. Toxin genes are coloured in blue and antitoxin genes in green. A single gene, STM4032 (in orange), separates the two TA modules. The promoter regions of the TA operons are shown as a blow-up. Putative transcriptional start sites are shown as broken arrows. Start sites of the first gene in the TA operons are shown in green bold letters. Putative −10 and −35 sequences are boxed. Palindromic sequences that are putative antitoxin binding sites are shown as opposing arrows.

The article "A Toxin-Antitoxin Module of Salmonella Promotes Virulence in Mice" was retracted in 2020. Reasons: manipulated images; duplicated images; concerns about the images.

### The toxin components of *sehAB* and *sehCD* are moderately toxic or non toxic for *Salmonella* grown in artificial media

To assess the putative functions of these modules, we expressed the predicted toxins in *E. coli* from an inducible promoter. The growth in Luria-Bertani (LB) broth of *E. coli* strains was measured over a period of 8 hours. A group of five proteins (group 1 in Figure 2A) exerted a strong bacteriostatic effect in E. coli. The expression of seven other putative toxins (group 2) only slightly attenuated bacterial growth, suggesting that these proteins are either not toxins or that their toxicity is limited in a heterologous expression system.

**Figure 2:** Effect of toxins and antitoxins on bacterial growth. Bacteria were grown at 37°C in LB broth and the optical density was monitored (**A** & **C**) or the colony forming units (CFU) were enumerated (**B**). (**A**) Effect of *Salmonella* toxins over-expression on *E. coli* growth. BL21(DE3) cells were transformed with an empty pDEST17 (ctrl) or derived plasmids carrying the putative *S.* Typhimurium toxin genes. Toxin expression was induced by adding 1 mM IPTG 2 hr after inoculation. Group 1: STM2954.1n, STM3516, STM3558, PSLT028. Group 2: STM1550, STM3033, STM3777, STM4031, STM4032.2N, STM4450, PSLT106. (**B** & **C**) Growth kinetics of wild-type (WT) and *sehAB* mutant strains of *S*. Typhimurium. When indicated, strains were complemented with pDEST49-derivative vectors for the expression of SehA, SehB or SehD under the control of the arabinose-inducible promoter.

Next, we focused our studies on TA modules present in all *Salmonella* strains capable of infecting warm-blooded animals (Figure 1A). More precisely, we targeted STM4031-STM4030.S and STM4032.2N-STM4033, which presented a close chromosomal location, being separated by a single unrelated gene, and encode transcripts on opposite chromosome strands (Figure 1B).

The article "A Toxin-Antitoxin Module of Salmonella Promotes Virulence in Mice" was retracted in 2020. Reasons: manipulated images; duplicated images; concerns about the images.

STM4031-4030.S encodes proteins presenting 40% and 46% identity with HigB and HigA from *E. coli* (Taxonomy ID 83333), respectively. The product of STM4032.2N presents 72% identity with HigB of *E. coli* (Taxonomy ID 561). While both STM4030.S and STM4033 products possess an HTH-XRE DNA binding domain that is found in type II antitoxins, they do not present significant shared similarity (7.7% identity). Likewise, the toxic components (STM4031 and STM4032.2N) show only 11.6% identity and none exerted strong toxicity in *E. coli* (Group 2 in Figure 2A). We renamed these TA gene locus *seh* (*Salmonella enterica* Hig-like) modules. Hence, STM4031-STM4030.S and STM4032.2N-STM4033 correspond to *sehAB* and *sehCD*, respectively (Figure 1).

We examined the chromosomal location and organization of *sehAB* and *sehCD* locus in several strains of *Salmonella*. A bioinformatics analysis revealed that *sehAB* and *sehCD* are not present in genomic islands, yet a cluster of genes similar to that found in S. Typhimurium was present in all strains of the species *enterica* (except *arizonae* in which *sehAB* is missing), (Figure S1). This cluster of genes has a conserved chromosomal location and is missing in the species *bongori*.

We generated various *S*. Typhimurium mutants of *sehAB* and *sehCD* and evaluated the impact of these deletions on bacterial growth. While deletion of the *higA* antitoxin gene in *Mycobacterium tuberculosis* [20], *Vibrio cholerae* [21] or *Pseudomonas aeruginosa* [22] is lethal, we were able to generate *Salmonella* mutants deleted of either antitoxin gene. A mutant deleted of the gene coding for the SehB antitoxin (Δ*sehB*) formed tiny colonies on agar plates and grew slower than the wild-type strain in LB broth, while over-expression of the SehA toxin limited the growth of the wild-type *S.* Typhimurium strain (Figure 2B). No growth change was observed in absence of the toxin (Δ*sehA*) or in absence of the module (Δ*sehAB*). Thus, the bacteriostatic effect was observed where there was excess of toxin or in the absence of antitoxin, suggesting that SehAB functions as a toxin-antitoxin system. The growth defect of *ΔsehB* was complemented by plasmid for the expression of the antitoxin (pSehB) under the control of the *ara* promoter (Figure 2C). Of note this complementation was also observed in absence of arabinose probably because of low level of expression. Remarkably, a Δ*sehB* mutant over-expressing SehB grew faster and to a higher density than the wild-type strain (Figure 2C). This suggests that SehA limits the growth of *S*. Typhimurium in a way that might reflect the topological organization of the *sehAB* operon in which the SehA toxin is transcribed first and may therefore be more abundant than its cognate antitoxin. However, wild-type and Δ*sehA* strains had similar growth curves (Figure 2B) and a Δ*sehA* strain over-grew when its cognate antitoxin was over-expressed (Figure S2A). These data indicate that the SehB antitoxin not only neutralizes its cognate toxin, but is also beneficial for *Salmonella* growth in a toxin-independent manner.

The article "A Toxin-Antitoxin Module of Salmonella Promotes Virulence in Mice" was retracted in 2020. Reasons: manipulated images; duplicated images; concerns about the images.

The Δ*sehC*, Δ*sehD* and Δ*sehCD* mutant strains were indistinguishable from the parental strain indicating that the toxin component is not limiting bacterial growth (Figure S2B). However, over-expression of the SehD antitoxin was able to partially complement for the absence of SehB (Figure 2C). Therefore we tested if SehD supported the growth of a Δ*sehB* mutant, as this mutant was unexpectedly viable. This hypothesis was tested by deleting *sehD* in a Δ*sehB* strain. We obtained a viable mutant deleted of both antitoxin genes (Δ*sehB* Δ*sehD*) indicating that SehD is not required for *Salmonella* growth in absence of SehB and *vice versa*. Altogether, these results indicate that, in LB broth, the SehC toxin does not impair *S*. Typhimurium growth while SehA exerts a non-lethal toxicity that is neutralized by its cognate antitoxin.

### The antitoxin components of SehAB and SehCD repress their own transcription

We undertook a biochemical and biophysical characterization of SehAB and SehCD and checked whether these modules regulate their own expression by binding palindromic sequences in their promoter region as expected for type II TA systems [2]. We found two perfect or near perfect palindromic sequences in the *sehAB* and *sehCD* promoter regions, which overlap with the putative −35 and/or −10 sequences (Figure 1B). To test whether SehB and SehD repress the expression of their operons, we generated plasmid-based transcriptional reporters by fusing the *sehAB* and *sehCD* promoter regions to the *gfp*mut3a gene. Bacteria carrying these reporter constructs were grown in LB broth and the fluorescence level of bacteria was monitored by flow cytometry [23]. The expressions of the *sehAB*-*gfp* and *sehCD*-*gfp* transcriptional fusions were 50- and 10-fold increased, respectively, in the absence of their relevant antitoxin or module, whereas the absence of the cognate toxin alone did not modify GFP expression (Figure 3A). By combining transcriptional reporters, mutants and plasmids we found that SehB does not repress SehCD expression and *vice versa* (Figure S3). This was predictable given that palindromic sequences and the nucleotide sequences between the palindromes are distinct in *sehAB* and *sehCD* promoter regions (Figure 1B).

The article "A Toxin-Antitoxin Module of Salmonella Promotes Virulence in Mice" was retracted in 2020. Reasons: manipulated images; duplicated images; concerns about the images.

**Figure 3:** SehB and SehD antitoxins bind to their promoter region. (**A**) Expressions of *sehAB*-*gfp* and *sehCD*-*gfp* are de-repressed in absence of their relevant antitoxin. *S*. Typhimurium wild-type (WT) and various mutant strains carrying a transcriptional fusion *sehAB*-*gfp* or *sehCD*-*gfp* were grown in LB broth and samples were taken at 4 hr post-inoculation. The relative fluorescence intensity of bacteria was determined by flow cytometry. Between 5000 and 10.000 bacteria were analysed to calculate the mean GFP/bacterium. (**B**) The SehB antitoxin binds specifically to its promoter region. An Electrophoretic mobility shift assay was carried out by incubating 100 ng PCR products covering *sehAB* (22.5 nM) or STM3558-59 (20 nM) promoter regions and increasing amounts [His]_6_-SehB as indicated. The complexes were separated on 6% polyacrylamide gels and DNA stained. (**C**) Surface Plasmon Resonance analysis of the binding of purified SehB to immobilized dsDNA. Sensorgrams for the interaction of various concentrations of SehB (62.5, 125, 250, 500 and 1000 nM) with immobilized DNA (300 resonance units). Inset shows fitting curve for equilibrium binding that resulted in a K_D_ of 150±30 nM. (**D**) SehA is pulled-down by SehB. Purified GST or GST-SehB were incubated with an extract a *E. coli* cells over-expressing [His]_6_-SehA or [His]_6_-SehC. After washing, proteins bound to glutathione-beads were separated by SDS-PAGE and analysed either by Coomassie blue staining of the acrylamide gel or by electrotransfer on a PVDF membrane and Western Blotting using an anti-[His]_6_ antibody.

Next, we investigated if the antitoxin-mediated repression was due to direct binding of antitoxins to their promoter regions [2]. We performed electrophoresis mobility shift assays (EMSA) using purified [His]_6_-tagged versions of antitoxins and PCR products covering the promoter regions of the operons. Both antitoxins specifically bound to their respective *seh* promoter region in a concentration-dependent manner (Figures 3B and S4), but not to the STM3559-58 promoter region used as a control. SehB and SehD bound with high affinity since the formation of the promoter DNA-antitoxin complexes reached a plateau below 250 and 500 nM, respectively. By comparison, the binding saturation of *M. tuberculosis* HigA to its promoter required one hundred times more concentrated protein [20]. We used Surface Plasmon Resonance to better characterize the interaction between SehB and its promoter region. We immobilized a biotinylated DNA oligomer corresponding to the sequence of the first palindrome of the *sehAB* promoter on a streptavidin chip, and assayed the binding of purified SehB. We measured a K_D_ of 150±30 nM, thus confirming the high affinity of SehB for this palindromic sequence (Figure 3C).

The article "A Toxin-Antitoxin Module of Salmonella Promotes Virulence in Mice" was retracted in 2020. Reasons: manipulated images; duplicated images; concerns about the images.

Using size-exclusion chromatography coupled with online multiangle laser light scattering (ultra-violet light absorbance and refractive index detectors) we characterized the formation of complexes between the SehAB proteins and the DNA palindromic sequence. We observed that purified SehB formed a stable dimer at 32 kDa (theoretical mass 31.4 kDa) (Figure S5). In the presence of DNA, we observed a mass of 34.4 kDa for the antitoxin dimer, of 14.6 KDa (theoretical mass 14.0 kDa) for the dsDNA, and of 49 kDa for the complex. We found that purified SehA formed a tetramer and higher aggregate but we were unsuccessful at reconstituting a toxin-antitoxin or a ternary complex using these purified proteins. However, GST-SehB specifically pulled-down [His]_6_-SehA from a bacterial extract (Figure 3D). This indicates that proteins of the *sehAB* module are capable of interacting. We concluded that repression of *sehAB* transcription is mediated by the binding of either the SehAB toxin-antitoxin complex or the SehB homo-dimer to its promoter region.

### Transcription of the *sehAB* locus is modulated by environmental conditions

Antitoxins of type II systems are believed to be more prone to proteolytic degradation than their cognate toxins. It results in increased availability of toxins as well as increased transcription of TA operons. In order to compare the stability of SehA and SehB, we constructed *S.* Typhimurium strains chromosomally expressing either SehA-3XFLAG or SehB-3XFLAG. These strains were grown for 6 hours in minimal medium after which protein synthesis was blocked with chloramphenicol. The level of pre-existing FLAG-tagged SehA and SehB was monitored during 60 min by Western Blotting. While the SehA toxin was remarkably stable, we noticed a marked decrease in SehB antitoxin signal during this period of time (Figure 4A). This result shows that SehB is labile as compared to SehA. Next, we determined if the transcriptional activity of *seh* loci is modulated in response to conditions encountered during interactions with animal cells. Wild-type *S*. Typhimurium and *sehAB* locus mutant strains carrying *sehAB-gfp* or *sehCD-gfp* transcriptional reporters were used to infect RAW 264.7 mouse macrophages. These strains were also grown in minimal medium, which is known to induce the expression of genes necessary for intracellular survival/replication [24]. As control, we used a transcriptional reporter for *sifA*, which is required for intracellular replication and is up-regulated in these growth conditions (Figure 3B). As compared to bacteria grown in LB broth, fluorescence resulting from expression of *sehAB*-*gfp* in wild-type *Salmonella* increased significantly both in minimal medium (4.3 times) and in macrophages (3 times) (Figure 4B). We observed a very similar profile of transcriptional activity in the absence of SehA, thus confirming that the toxin does not play a significant role in the regulation of the operon activity. As shown previously (Figure 3A), the transcriptional activity of *sehAB* increased dramatically in the absence of the antitoxin (Δ*sehB*) or the full module (Δ*sehAB*). Yet, in spite of the strong de-repression due to the absence of the antitoxin, *sehAB-gfp* expression was still approximately 1.5 times more increased in mutant strains grown in minimal medium as compared to LB broth. These results suggest that in addition of the repression mediated by the antitoxin, the transcriptional activity of the *sehAB* promoter is controlled by additional regulatory elements which are at least partly dependent on environmental conditions. The expression of *sehCD-gfp* increased about three and 1.5 times in bacteria grown in minimal medium or in macrophages, respectively (Figure 4C). The *sehCD* promoter was insensitive to the absence of either or both SehAB proteins. We concluded that the *sehAB* loci responds to conditions encountered inside host cells, therefore suggesting this module might influence the intracellular growth of *S*. Typhimurium.

The article "A Toxin-Antitoxin Module of Salmonella Promotes Virulence in Mice" was retracted in 2020. Reasons: manipulated images; duplicated images; concerns about the images.

**Figure 4:** Regulation of *sehAB* and *sehCD* promoters and role of SehAB proteins in intracellular replication. (**A**) SehB is prone to degradation. Strains expressing chromosomally SehB-3XFLAG or SehA-3XFLAG were grown for 6 hours in minimal medium. 100 µg/ml chloramphenicol was then added and samples were taken at the indicated times. The presence of remaining SehA and SehB was analysed by Western Blotting using an anti-FLAG antibody. (**B** & **C**) Expression of *sehAB*-*gfp* is de-repressed in minimal medium and inside mouse macrophages. Wild-type (WT) *S*. Typhimurium and *sehAB* mutant strains carrying the transcriptional fusion *sifA-gfp*, *sehAB-gfp* or *sehCD-gfp* were grown in LB broth, minimal medium (MM) or inside RAW 264.7 mouse macrophages. Bacteria were collected at 4 (LB) or 16 (MM) hours post-inoculation or extracted from macrophages 16 hours post-infection. The relative GFP fluorescence intensity of bacteria was determined by flow cytometry. (**D**) *sehAB* is dispensable for intracellular replication. C57BL/6 bone marrow-derived macrophages were infected with wild-type (WT) or various *sehAB* mutant strains. Δ*sifA* and Δ*ssaV* strains were used as controls. Cells were lysed at 2, 8 and 14 hr post-infection for enumeration of intracellular bacteria. A representative experiment is shown. The graph values are the mean colony forming units (CFU) per well ± SD of triplicates. The “fold replication” for the presented experiment was calculated as a ratio of the intracellular bacteria between 14 and 2 hr. The “normalized replication” represent the fold increase calculated as a ratio of the intracellular bacteria between 16 and 2 hr and normalized to that of the wild-type strain (100%). Values are means ± SD of 3 independent experiments.

### *sehAB* and *sehCD* are dispensable for intracellular replication

Cell lines and primary cells were used to investigate the potential role of *seh* modules in intracellular replication of *Salmonella*. Bone marrow-derived macrophages (BMM) were infected with *sehAB* mutant strains and the numbers of intracellular bacteria were determined at 2, 8 and 14 hours post-infection. We also calculated the relative fold increase of intracellular bacteria between 2 and 14 h post-infection with respect to the wild-type strain (100%). As expected, we observed at 14 hours post-infection a dramatic replication defect for the control Δ*ssaV* mutant strain [25] (Figure 4D). Bacteria deleted of *sehB* or *sifA* [26] presented a moderate intracellular replication defect (relative fold increase of 48±6% and 43±3%, respectively). Mutants deleted for *sehA* or the full module (Δ*sehAB*) replicated similar to the wild-type strain, indicating that *sehAB* is dispensable for replication inside BMM.

The intracellular replication of *seh* mutants was also tested in human HeLa cells and RAW 264.7 mouse macrophages. We also observed in these cell lines a moderate intracellular replication defect for the Δ*sehB* mutant while deletion of either or both *sehCD* genes had no effect (Figure S6A). Strains over-expressing either antitoxin replicated more than twice as much as the control, whether the absence or presence of their cognate toxin or module (Figure S7).

Next we tested whether the replication defect of a Δ*sehB* antitoxin mutant could be attributed, at least in part, to a direct toxic effect of the SehA toxin on eukaryotic cells. Infected macrophages were stained with fluorescent markers for death and early apoptosis and analyzed by flow cytometry. Infection by *Salmonella* increased the percentage of cells positive for both markers from about 1 to 10%, no matter which strain was used (Figure S8). These results indicate that the presence of high level of free SehA toxin in *Salmonella* does not impact the viability of infected cells.

The article "A Toxin-Antitoxin Module of Salmonella Promotes Virulence in Mice" was retracted in 2020. Reasons: manipulated images; duplicated images; concerns about the images.

We concluded that i) SehAB and SehCD are dispensable for intracellular replication, ii) Over-expression of either antitoxin confers to *Salmonella* an intracellular hyper-replicative phenotype similar to that observed in LB broth, and iii) The moderate intracellular growth defect of the Δ*sehB* strain is likely nonspecific and rather results from a general growth defect for this strain.

### SehAB is a virulence factor in perorally inoculated mice

We compared the virulence of wild-type and *seh* mutant strains in mice by performing mixed infections. As controls, we again used the Δ*sifA* and Δ*ssaV* strains that respectively, are moderately and highly attenuated in this model [27]–[29]. Groups of C57BL/6 mice were inoculated intraperitoneally with different two strain combinations (1∶1 mix) and bacteria were recovered from mouse spleens after 2 days to determine the competitive index (CI) [30]. We found that the Δ*sehB* antitoxin mutant is highly attenuated with respect to the wild-type strain (CI = 0.02±0.01). Remarkably, this attenuation is more pronounced and similar to that observed with the Δ*sifA* (CI = 0.16±0.05) and Δ*ssaV* strains (CI = 0.01±0.003) (Figure 5A). Complementation with a plasmid for the expression of SehB allowed the Δ*sehB* mutant to recover virulence (CI = 0.75±0.2), while the Δ*sehA* and Δ*sehAB* mutant strains displayed a wild-type level of virulence. These results demonstrate that, while the *sehAB* module is dispensable for systemic infection, SehA exerts *in vivo* a very strong toxic action that is neutralized by its cognate antitoxin (Figure 5A).

**Figure 5:** *sehAB* is transiently involved in Salmonella virulence upon peroral inoculation. Mice were inoculated intraperitoneally (**A**) or perorally (**B** & **C**) with a 1∶1 mixture of two *Salmonella* strains as indicated. C57BL/6 mice we used, except for panel C for which 129S2 and C57BL/6 mice were infected as indicated. Spleens were harvested two days (**A**), five days (**B**) or at various times (**C**) post-inoculation and bacteria were enumerated. The lowest and highest total CFU/organ in each group of CI were in (**B**) WT *versus* : Δ*sehAB*, 8.7×10^5^–2.3×10^7^; Δ*sehB*, 2.3×10^5^–1.9×10^8^; Δ*sehA*, 4.3×10^3^–2.5×10^7^; Δ*sehAB* pSehAB, 5.2×10^4^–1.3×10^8^; Δ*sehAB* Δ*sehCD*, 6×10^5^–1.4×10^7^; (**C**) WT *versus* Δ*sehAB* in 129S2: Day 5, 2.8×10^3^-1.3×10^4^; day 14, 3.6×10^4^-6×10^4^; day 18, 2.5×10^4^-1.2×10^6^; in C57BL/6: 8.7×10^5^-6.2×10^6^. Each symbol represents a mouse and horizontal bars correspond to the means ± SD. A one-sample *t*-test was used to determine whether a CI was significantly different of one, and unpaired *t*-tests to determine whether two values were significantly different. *P*-values: ns, not significant; *, *P*<0.05; **, *P<*0.01; ***, *P*<0.0005.

The article "A Toxin-Antitoxin Module of Salmonella Promotes Virulence in Mice" was retracted in 2020. Reasons: manipulated images; duplicated images; concerns about the images.

Next, we tested if this module could play a role in mice inoculated by the natural route. We found that by peroral inoculation, a strain deleted of *sehB* also presents a strong virulence defect (CI = 0.16±0.06) while bacteria deleted of the toxin are unaffected (CI∼1) (Figure 5B). Interestingly, the Δ*sehAB* strain is significantly attenuated (CI∼0.50) (Figure 5B and 5C) but complemented by a plasmid expressing SehAB under its natural promoter (Figure 5B). We also examined the role of SehAB in 129S2 mice carrying wild-type alleles of Nramp1. 129S2 mice have been used to develop a model of persistent *S*. Typhimurium infection [31], [32] and we took advantage of the prolonged survival of *Salmonella*-infected 129S2 mice to analyze the evolution of the CI with time. At five days post-inoculation, a Δ*sehAB* strain presented in 129S2 mice an attenuation (CI = 0.64±0.24) similar to that observed in C57BL/6 mice (Figure 5C). Surprisingly, this value did not decrease to a great extent with time but rather tended to reach a plateau (CI = 0.41±0.05 at day eighteen post-inoculation, Figure 5C). These results suggest that after an initial deficiency in establishing an infection by the natural route, the Δ*sehAB* mutant is able to persist as well as the wild-type strain. It confirms that *sehAB* does not play a significant role in the systemic infection. Rather, this module is involved in the early phase of peroral infection.

Strains deleted of *sehAB* or of both *sehAB* and *sehCD* were not significantly different in their virulence attenuation when given perorally to C57BL/6 (Figure 5B). This indicates that the *sehCD* module, whose toxin does not seem to be active in mice (Δ*sehD* in Figure 5A), does not contribute significantly to *Salmonella* virulence in the mouse model.

### *sehAB* is highly transcribed in mesenteric lymph nodes and is required for survival of *Salmonella* in these organs

The attenuation of a Δ*sehAB* mutant suggested that upon peroral inoculation *Salmonella* encounters conditions favouring the enhanced transcription of the *sehAB* locus. To confirm this, we inoculated mice with wild-type *S*. Typhimurium carrying a transcriptional reporter for *sehAB* (*sehAB-gfp*). Bacteria extracted from various organs were examined for the expression of GFP by flow cytometry and compared to reference strains grown in LB broth. Most *Salmonella* extracted from the mesenteric lymph nodes (MLN) of perorally inoculated mice showed GFP fluorescence levels (blue curve, Figure 6A) that were slightly higher than that of wild-type *S.* Typhimurium grown in LB broth (green curve, Figure 6A). This indicates that the majority of bacteria in the MLNS exhibit slightly higher expression of *sehAB*. Yet, we also observed in MLNs a second population with a mean GFP fluorescence similar to that observed for the Δ*sehB* strain grown in LB broth (red curve, Figure 6A). This population, hereafter referred to as GFP^high^ bacteria, corresponded to *Salmonella* in which expression of *sehAB* is de-repressed. This GFP^high^ population although not exceeding 5% of the total *Salmonella* population, was however significantly more prevalent in spleens and MLNs of mice inoculated *via* the peroral route (Figure 6B). The mean fluorescence of total bacteria was also significantly increased in populations extracted from perorally but not from intraperitoneally inoculated mice, when compared to bacteria grown in LB broth (Figure 6C). Finally, in perorally inoculated mice, the mean fluorescence of GFP^high^ bacteria was significantly higher in *Salmonella* extracted form MLNs in comparison to their corresponding spleens (Figure 6C). Considering that having crossed the intestinal barrier the bacteria will reach the MLNs before the spleen [33], these results indicate that activation of the *sehAB* module is an early event in the process of infection through oral ingestion. To further emphasise this point we also analysed the consequences of the deletion of *sehAB* on the virulence attenuation of bacteria present in various organs. We found that the CI of wild-type *versus* Δ*sehAB* strains is much lower in MLNs (0.05±0.03) as compared to the spleen (0.51±0.19) and the liver (0.32±0.02) (Figure 6D). These results reveal that *sehAB* is especially important for the survival of bacteria in MLNs.

The article "A Toxin-Antitoxin Module of Salmonella Promotes Virulence in Mice" was retracted in 2020. Reasons: manipulated images; duplicated images; concerns about the images.

**Figure 6:** *sehAB* is highly transcribed in a small population of bacteria upon peroral inoculation. (**A**–**C**) C57BL/6 mice were inoculated intraperitoneally or perorally as indicated with wild-type *S*. Typhimurium carrying a transcriptional fusion *sehAB-gfp*. The relative GFP fluorescence intensity of bacteria extracted from the spleen or MLNs was determined by flow cytometry. Between 5000 and 10.000 bacteria were analysed for each sample. (**A**) A small population of *Salmonella* extracted from infected mice are highly fluorescent. Bacteria were extracted from MLNs of a mouse five days post-peroral inoculation. Bacteria were analyzed by flow cytometry for GFP fluorescence (blue) and compared to bacteria used for the inoculation (green) and, as control, with a Δ*sehB* strain (red). Bacteria extracted from MLNs contain a population expressing a high level of GFP (GFP^high^). (**B**) The percentage of GFP^high^ bacteria is significantly higher in mice inoculated perorally *versus* intraperitoneally. Bacteria were extracted from spleens or MLNs of mice inoculated intraperitoneally or perorally and the percentages of GFP^high^ bacteria were determined. (**C**) The mean GFP fluorescence of total and GFP^high^ bacteria is significantly increased in bacteria extracted from perorally inoculated mice and significantly higher in MLN *versus* spleen. The mean GFP fluorescence was normalized to that of bacteria used for inoculation. (**D**) The CI of wild-type versus Δ*sehAB* is lower for the population of bacteria extracted from MLNs. C57BL/6 mice were inoculated perorally with a 1∶1 mixture of wild-type and Δ*sehAB* strains. Spleen, liver, MLNs and the small intestine (S. I.) were collected five days post-inoculation and bacteria were enumerated. Each symbol represents a mouse, and horizontal bars correspond to the means ± SD. The lowest and highest total CFU/organ in each group of CI were in : spleen, 8.8×10^6^-7.5×10^7^; Liver, 7×10^7^-2.1×10^8^; MLNs, 6.5×10^4^-1.9×10^5^; S. I., 7.1×10^5^-5×10^6^. (**B**–**D**) A one-sample *t*-test was used to determine whether a value was significantly different of one and an unpaired *t*-tests to determine whether two values were significantly different. *P*-values: ns, not significant; *, *P*<0.05; **, *P<*0.01; ***, *P*<0.0005.

## Discussion

Type II TA modules are inhibitors of translation that induce bacterial dormancy. Being in a dormant state helps bacteria to survive harmful environments. For example, type II TA modules favour resistance to antibiotics [1]. This study presents evidence that virulent strains of *Salmonella* possess multiple TA systems and shows that one of these is beneficial in the early phase of infection by the natural route.

We ascertained the presence of eleven type II TA modules in *S.* Typhimurium and examined the presence of homologous genes across Salmonellae. A heatmap generated using both strains and TA gene modules highlighted a set of four TA that are found across serovars of *S. enterica* infecting warm-blooded animals. In contrast, non-pathogenic species and strains of *S. enterica*, which are associated with cold-blooded animals, possess no or low numbers of TA modules found in *S* Typhimurium, respectively. Interestingly, previous data extracted from a transcriptional profile of intracellular *S*. Typhimurium [34] showed that the expression of the eleven TA modules is induced during infection of mouse macrophages, thus highlighting the possible involvement of these modules during the interaction with host cells.

The article "A Toxin-Antitoxin Module of Salmonella Promotes Virulence in Mice" was retracted in 2020. Reasons: manipulated images; duplicated images; concerns about the images.

It is important to note that the present study did neither perform an exhaustive review of TA modules in *Salmonellae*, nor investigate whether the non-pathogenic species *S. bongori* or strains infecting cold-blooded animals have specific TA module repertoires. It is very likely that other TA systems exist and will be discovered as illustrated by the recently published study by Slattery et al. [35]

These TA operons, which are part of the prokaryotic mobilome [36], are likely to have been acquired by horizontal transfer and positively selected because of their advantage for pathogenesis. Strikingly, the *sehAB* and *sehCD* loci delineate a gene cluster that has a conserved location on chromosomes of various virulent strains of *S. enterica*. This suggests that a common ancestor of the *enterica* species has acquired this cluster as a block, and provides further indication that these TA modules play a role in virulence.

We found that a mutant deleted of *sehAB* is attenuated for virulence in mice inoculated perorally but fully virulent in mice inoculated intraperitoneally. This is reminiscent to what has been observed for the SP1-encoded type three secretion system [37], which helps *Salmonella* to cross the intestinal barrier. Thus, *sehAB* is likely to play a role in an early step of the infection process that is temporally localized between the arrival of the bacterium in the stomach and the triggering of a systemic infection. Interestingly, the CI in spleens of perorally inoculated mice was the same at 5 and 18 days post-infection, thus confirming that *sehAB* plays a transient role and is not involved in the systemic phase of the infection. The stomach and the gut are aggressive environments in which the activation of *sehAB* might favour persistence. Peyer's patches are preferential sites for *Salmonella* to cross the intestinal barrier [38], [39]. MLNs into which Peyer's patches are drained are central sites for the induction of the mucosal immune response and possess an important antibacterial arsenal. Thus, another possibility is that *sehAB* helps *Salmonella* to survive the biochemical stresses (NO, antibacterial peptide…) and/or the innate immune cellular defences present in the subepithelial environment. Indeed, this possibility is supported by the presence of *Salmonella* with high *sehAB* promoter activity in MLNs and by the low CI of a Δ*sehAB* mutant in these peripheral lymphoid organs. The association of these data suggests that an up-regulation of the *sehAB* promoter helps *Salmonella* to survive the detrimental environment of the MLNs.

The article "A Toxin-Antitoxin Module of Salmonella Promotes Virulence in Mice" was retracted in 2020. Reasons: manipulated images; duplicated images; concerns about the images.

Five days post-inoculation we detected in MLNs a maximum of five percent of GFP^high^ bacteria. We cannot exclude the possibility that the activation of *sehAB* occurs earlier and in a larger part of the bacterial population. However, our attempts to detect fluorescent bacteria in mice at earlier times post-inoculation were unsuccessful because the number of bacteria present in the various organs was too low.

The HigB toxin of *E. coli* K12 cleaves mRNAs positioned at the ribosomal A-site and stops translation [40]. The mechanism of action of the SehA toxin is unknown but, considering it shares 40% identity with HigB, these toxins are likely to have similar targets. However, our results indicate that SehA activity is dependent on an additional mechanism. Indeed, a Δ*sehB* strain, which expresses a high level of free toxin, presents only a partial growth defect in LB broth or in cultured cells but is severely impaired for virulence in the mouse model. Interestingly, a previous screen performed in a mouse model selected STM4030 (*sehB*) among the most important genes for virulence [41]. Altogether, this indicates that the toxin itself is necessary but not sufficient to limit bacterial growth and that an additional factor synergizes with SehA activity under conditions of mouse infection. This might be an activator/inhibitor factor whose association/dissociation with the toxin is controlled by environmental conditions encountered in mice. This factor is operational in intraperitoneally inoculated mice although a Δ*sehAB* remains fully virulent under these conditions of infection. Overall it suggests that activation of the SehA toxin and transcription of the *sehAB* locus are not triggered by the same environmental conditions.

In general toxins and antitoxins form hetero-oligomers that are toxin-inhibiting complexes that can bind their promoter region [42], [43]. We could not reconstitute a SehAB toxin-antitoxin complex using purified proteins. In addition, we observed an aggregation of purified SehA, which might result from non-native folding and could explain its lack of interaction with the antitoxin. Nevertheless SehA was specifically pulled-down by SehB from a bacterial extract, indicating that SehA and SehB are likely to form a canonical type II TA complex.

Stress conditions leading to the de-repression of *sehAB* are poorly mimicked in cultured cells. This is shown by the limited activation of the *sehAB* promoter and by the absence of growth defect in the Δ*sehAB* mutant. This suggests that this locus does not support the survival/replication of intracellular bacteria. Another possibility is that cultured cells and bone marrow-derived macrophages are not representative of cell types encountered by *Salmonella* during the early phase after oral inoculation. *sehAB* might help the bacterium to survive bactericidal activity mediated by immune cells that are recruited to the infection sites. Supporting this observation is the fact that *Salmonella* are not killed and can survive in dendritic cells. Of note, this survival is independent of virulence factors known to be important in macrophages [44].

The article "A Toxin-Antitoxin Module of Salmonella Promotes Virulence in Mice" was retracted in 2020. Reasons: manipulated images; duplicated images; concerns about the images.

We could not find any phenotype associated with *sehCD*. Nevertheless, this locus like *sehAB*, is conserved among pathogenic strains of *Salmonella enterica* indicating its importance for the general fitness of *Salmonella*. The *sehCD* locus might for example, be necessary for interactions with another warm-blooded *Salmonella* host.

The present study supports the idea that type II TA modules sustain *Salmonella* virulence. Likewise, *M. tuberculosis* contains many more TA systems than the saprophytic *M. smegmatis*, leading to the suggestion that TA modules play a role in virulence by supporting the long-term dormancy of the pathogen in macrophages [45]. TA systems of extra-intestinal pathogenic *E. coli* have recently been shown to also impact the persistence of bacteria within host tissues [12]. Thus, it is more and more apparent that TA systems are important elements in the virulence of bacterial pathogens. The next challenge will be to understand the signalling and biochemical processes supporting the full activation of the SehA toxin and when and where the conditions necessary for this activation are encountered in the course of oral inoculation. Finally, it will be essential to evaluate the importance and role of other type II TA modules in *Salmonella* pathogenicity.

## Materials and Methods

### Ethic statement

Animal experimentation was conducted in strict accordance with good animal practice as defined by the French animal welfare bodies (Law 87–848 dated 19 October 1987 modified by Decree 2001-464 and Decree 2001-131 relative to European Convention, EEC Directive 86/609). All animal work was approved by the Direction Départementale des Services Vétérinaires des Bouches du Rhône (authorization number 13.118 to S.M.).

### Bacterial strains and growth conditions

Bacterial strains and plasmids used in this study are listed in Table S1 in Text S1. Strains were cultured in LB broth (Difco) or minimal medium (M9, glycerol 0.2%, MgSO_4_ 1 mM, CaCl_2_ 200 mM, thiamine 1 mg/ml, casamino acids 1 mg/ml. Ampicillin (50 µg/ml), kanamycin (50 µg/ml), tetracycline (10 µg/ml) and chloramphenicol (50 µg/ml) were added when required. Bacterial suspensions were prepared from overnight LB broth cultures that were centrifuged and resuspended in fresh LB broth or minimal medium to an OD_600_ of 1. Then, 250 ml-flasks containing 50 ml of LB broth or minimal medium were inoculated with 1 ml of the bacterial suspensions and incubated at 37°C in a shaking incubator at 200 rpm.

The article "A Toxin-Antitoxin Module of Salmonella Promotes Virulence in Mice" was retracted in 2020. Reasons: manipulated images; duplicated images; concerns about the images.

### Toxin-antitoxin databases and identification

Using RASTA webtool and standard BLASTP, we searched the *S*. Typhimurium genome for sequences coding for toxins and antitoxins belonging to the seven known type II TA super families: vapBC, relEB, parED, mazEF, phd-doc, ccdAB and higAB. In addition, we used others type II toxin-antitoxin sequences described for *E. coli* [2] (yafNO, hicAB, yefMyoeB, mqsRA, chpBIchpBK, rnlAB). For TA identification, the protein set from a whole genome was first arranged by genome coordinates. Each protein in our TA databases was then used in a BLASTP query. A hit was defined as a match to a query protein with an E-value threshold of 10^−5^, which should cover at least 70% of the TA with more than 30% identity. Lastly, a TA module was recognized if two contiguous proteins in the genome were possible toxin and antitoxin as suggested by the results of a BLASTP. In addition to BLASTP, we used the TBLASTN algorithm to search for the presence of toxin and antitoxin genes. Genomic locations of TA modules encoded by *Salmonella* sequenced strains were obtained from NCBI.

### Construction of mutant strains

Non-polar gene-deletion mutants were generated by the lambda Red recombinase system [46], using gene-specific primer pairs to amplify pKD4 kanamycin or pKD3 chloramphenicol resistance genes as shown in Table S2 in Text in Text S1. *Salmonella* mutants were transformed with the pCP20 plasmid to excise the antibiotic cassette. This excision was performed for the Δ*sehAB* mutant, which was then transformed with pK3-SehAB for the expression of SehAB under its natural promoter, and for *sehA*::3XFLAG and *sehB*::3XFLAG. Gene deletions were checked by PCR.

### Construction of plasmids

The *sehAB-gfp* and *sehCD-gfp* transcriptional fusions were generated by cloning PCR products corresponding to the respective promoter regions into pFPV25 [47] (see primers in Table S2 in Text S1). These PCR products were digested with EcoRI and BamHI and ligated to pFPV25 digested with the same enzymes. For *E. coli* expression, PCR products corresponding to *Salmonella* toxins were cloned in pDEST-17 using the Gateway system (Invitrogen, Ltd., Paisley, U.K.). *sehB* and *sehD* antitoxin genes were cloned both into pBAD-DEST49 and pMPM-K6. For pMPM-K6, primers contained the NcoI (5′)/HindIII (3′) restriction sites. The resulting PCR products were digested with NcoI and HindIII and ligated into pMPM-K6 [48] digested with the same restriction enzymes, generating the plasmids pK6-SehB and pK6-SehD. These plasmids contain the antitoxin genes under an arabinose inducible promoter. The *sehAB* locus was cloned in the pMPM-K3 plasmid for the expression of SehAB with its own promoter. The PCR product resulting from the amplification of chromosomal DNA of 12023 with the primers STA1T-EcoRI-5 and STA1T-HINDIII-3 was digested with HindIII and ligated into pMPM-K3 previously digested with SmaI-HindIII, generating the pK3-SehAB. All constructs were confirmed by DNA sequencing. Plasmids used in this study are listed in Table S1 in Text S1.

The article "A Toxin-Antitoxin Module of Salmonella Promotes Virulence in Mice" was retracted in 2020. Reasons: manipulated images; duplicated images; concerns about the images.

### Electrophoretic mobility shift assay (EMSA)

EMSA experiments were performed as described previously [49]. PCR products corresponding to *sehAB* and *sehCD* promoter regions were the same as used to generate *sehAB-gfp* and *sehCD-gfp*. These fragments (100 ng), were mixed with increasing concentrations of [His]_6_-tagged SehB or SehD in PBS/50% glycerol. They were incubated 30 min at room temperature and then separated by electrophoresis in 6% polyacrylamide gels in Tris-borate-EDTA buffer. The DNA bands were visualized by staining with ethidium bromide.

### Eukaryotic cells and culture conditions

RAW 264.7 and HeLa cell lines were grown in DMEM (GibcoBRL) supplemented with 10% foetal calf serum (FCS; GibcoBRL), 2 mM nonessential amino acids, and glutamine (GibcoBRL) at 37°C in 5% CO_2_.

### Bacterial infection and replication assays

Bone marrow-derived macrophages, HeLa and RAW 264.7 macrophage were grown, infected and treated as previously described [50].

### Analysis of SehAB proteins degradation and western blot analysis

Bacteria expressing SehA-3XFLAG or SehB-3XFLAG from the chromosome were grown during 6 h in minimal medium. Then, protein synthesis was stopped by addition of 100 µg/ml chloramphenicol, and samples were removed at the indicated time points. SehAB proteins were detected by Western Blotting using a monoclonal anti FLAG-tag antibody (Sigma-Aldrich) and a polyclonal goat-anti mouse IgG HRP conjugate (Sigma–Aldrich).

### Competitive index

Eight- to ten-week-old C57BL/6 or 129S2 mice were inoculated intraperitoneally or perorally with equal amounts of two bacterial strains for a total of 10^5^ bacteria per mouse. The spleens were harvested 2 or 5 days after inoculation, as indicated, and homogenized. Bacteria were recovered and enumerated after plating a dilution series onto LB agar with the appropriate antibiotics. Competitive indexes (CI) were determined for each mouse [30]. The CI is defined as the ratio between the mutant and wild-type strains within the output (bacteria recovered from the mouse after infection) divided by their ratios within the input (initial inoculum). Statistical analyses were performed using Prism (GraphPad, San Diego, CA, USA).

The article "A Toxin-Antitoxin Module of Salmonella Promotes Virulence in Mice" was retracted in 2020. Reasons: manipulated images; duplicated images; concerns about the images.

### Flow cytometry analysis of bacteria extracted from synthetic medium, macrophages or mouse organs

Bacteria grown in synthetic medium (LB broth or MM) or extracted from infected cells or mouse organs were treated and analyzed by flow cytometry as previously described [23].

## Supporting Information

Figure S1 **Chromosomal location of** ***sehAB*** **and** ***sehCD*** **loci in different** ***Salmonella*** **strains en species.** This graph is a representation of the chromosomal region on either side of *sehAB* and *sehBC* loci. The genes are coloured function of their GC%. *sehAB* and *sehAB* are indicated in blue and red circles, respectively. This image was performed using http://www.xbase.ac.uk.
(TIFF)

Figure S2 **Effect of toxins and antitoxins on** ***Salmonella*** **growth.** Strains were grown in LB broth and optical density was monitored at 600 nm every hour. (**A**) Over-expression of SehB is beneficial for *Salmonella* growth even in absence of its cognate toxin (SehA). Growth kinetics of a Δ*sehA* mutant strain of *S*. Typhimurium over-expressing or not SehB. (**B**) The toxin component of SehCD does limit the growth of *Salmonella* in LB broth. Growth kinetics of wild-type (WT) and *sehCD* mutant strains of *S*. Typhimurium.
(TIFF)

Figure S3 **SehB does not repress** ***sehCD*** **expression and conversely.** Expression of *sehAB*-*gfp* is unaffected by the absence (**A**) or the over-expression (**B**) of SehD and *vice versa*. Wild-type *S*. Typhimurium (WT) (**A & B**) or antitoxin mutant strains (**A**) carrying a transcriptional reporter *sehAB-gfp* or *sehCD-gfp* and over-expressing SehB or SehD under the control of an *ara* promoter were grown in LB broth and the samples were taken at 4 hr post-inoculation. The relative fluorescence intensity of bacteria was determined by flow cytometry and used to calculate the mean GFP fluorescence/bacterium.
(TIFF)

Figure S4 **SehD binds to its promoter region.** Electrophoretic mobility shift assays were carried out by incubating 100 ng PCR products covering *sehCD* (16.9 nM) or STM3559-58 (20 nM) promoter regions and increasing amounts [His]_6_-SehD as indicated. The complexes were separated on 6% polyacrylamide gels and DNA stained.
(TIFF)

Figure S5 **Stoichiometry of the SehB-DNA complex.** Purified SehB was subjected to size-exclusion chromatography coupled to MALS/RI/UV detectors as described in the Supporting Information. The absorption at 280 nm of SehB without DNA (AT, red line) and with DNA (green line) and the molar mass (black line), derived from refractive index measurements, were plotted as a function of the elution time. Molar mass values at the absorption peaks are indicated, with those resulting from protein-conjugate analysis in parenthesis.
(TIFF)

Figure S6 ***sehAB*** **and** ***sehCD*** **are dispensable for replication in cultured cells.** Mouse RAW 264.7 macrophages (**A**) or human HeLa cells (**B**) were infected with wild-type (WT) or various *sehAB* or *sehCD* mutant strains. Δ*sifA* and Δ*ssaV* strains were used as controls. Cells were lysed at 2 and 16 hr post-infection for enumeration of intracellular bacteria. The values shown represent the fold increase calculated as a ratio of the intracellular bacteria between 16 and 2 hr and normalized to that of the wild-type strain (100%). Values are means ± SD of 3 independent experiments. One-way ANOVA and Tukey post-tests were used to determine whether the values were significantly different. *P*-values: ns, not significant; *, *P*<0.05; ***, *P*<0.0005.
(TIFF)

Figure S7 **SehB and SehD are beneficial for *S.* Typhimurium intracellular replication.** RAW 264.7 macrophages were infected with various bacteria. The values are the fold increase calculated as a ratio of the intracellular bacteria between 16 and 2 hr and normalized to that of the wild-type strain or control strain containing the empty vector (pDEST49). Arabinose was added to the medium 1 hr post-infection as indicated. Fold increase of wild-type (**A**) or Δ*sehB* mutant (**B**) strains over-expressing or not SehB or SehD. STM3559 and PSLT027 antitoxins were over-expressed as controls. (**C**) Fold increase of wild-type, Δ*sehA* and Δ*sehAB* mutant strains over-expressing or not SehB. (**D**) Fold increase of wild-type, Δ*sehC* and Δ*sehCD* mutant strains over-expressing or not SehD.
(TIFF)

Figure S8 ***sehAB*** **does not influence the viability of infected mouse macrophages.** Raw 264.7 cells were infected with wild-type or various *sehAB* mutant strains expressing GFP. Cells were infected at a MOI of 25 and for 30 min with bacteria grown overnight in minimal medium, fixed at 16 hours post-infection and labelled with fluorescent annexin V and Aqua Dead. Cells were analyzed by flow cytometry. The percentages of annexin V-positive, Aqua Dead-positive, double-positive and double-negative among GFP-positive cells are indicated (in red).
(TIFF)

Text S1 **Supporting protocols and tables.** Protocols for 1) Protein production for biochemical/biophysical studies; 2) Multiangle light scattering; 3) Surface Plasmon Resonance. Table S1: *Salmonella* strains and plasmids used in this study; Table S2: Oligonucleotides used in this study.
(DOCX)
